The article "A Preliminary Study on the Equivalence between Standing Back-Extension and Superman Training in Lumbar Multifidus Exercise" was retracted in 2023. Reasons: unreliable results or conclusions; lack of ethics approval or compliance; concerns about the data; concerns about the peer review.

# A Preliminary Study on the Equivalence between Standing Back-Extension and Superman Training in Lumbar Multifidus Exercise

**DOI:** 10.1155/2022/3677831

**Published:** 2022-03-23

**Authors:** Youyin Xu, Jianguang Wang, Junxian Wu

**Affiliations:** Department of Orthopedics, Civil Aviation General Hospital, Beijing 100123, China

## Abstract

**Objective:**

To explore the equivalence of an easier and more convenient lumbar multifidus (LM) muscle exercise pattern among standing back-extension, static standing, and superman training.

**Methods:**

A total of 26 healthy young volunteers were enrolled, including 14 males and 12 females, aged from 22 to 44 years with an average of 31.77 ± 7.06 years. Ultrasonography was used to measure the thickness of the left LM of the transverse process of the L5 vertebra during static standing, static prone decubitus, standing back-extension, and prone superman training. In this study, measurement data were expressed as Mean ± SD and compared using the *t*-test.

**Results:**

The left LM thickness of the L5 vertebra was 2.92 ± 0.46 cm during static standing and 2.78 ± 0.39 cm during static prone decubitus, showing no statistical difference between the two groups (*P* > 0.05). The left LM thickness of the L5 vertebra was 3.16 ± 0.51 cm during standing back-extension and 3.33 ± 0.41 cm during the prone superman training, indicating no statistical difference between the two groups (*P* > 0.05).

**Conclusions:**

There is no significant statistical difference in the LM thickness between static standing and static prone decubitus and between standing back-extension and prone superman training, indicating the equivalence of the two methods in LM exercise, providing a simpler and easier way for clinical exercise of lumbodorsal muscles.

## 1. Introduction

Low back pain (LBP) is a common condition in clinical diagnosis and treatment. According to foreign studies, the disease has a predilection for people aged 35-55, with a prevalence of 7.6%-37% among different populations [1, 2]. LBP refers to the pain, muscle tension, and rigidity in any part of the human body from the costal margin of the back to the buttocks fold, with or without symptoms of the lower extremities. It is a group of symptoms or syndromes represented by pain in the back and loin, with irregular and recurrent attacks. LBP can be classified into many categories, but usually, it is divided into acute, subacute, and chronic according to the duration of pain <6 weeks, 6-12 weeks, and >12 weeks, respectively [3]. Ninety percent of acute episodes can be cured within 6 weeks, whereas 62 percent of people develop chronic LBP after the first episode, with symptoms lasting more than a year [4].

At present, the main methods to treat LBP include medicine, correction of biomechanics, physiotherapy, manipulation therapy, exercise training, gymnastics ball, and sling system. Of them, exercise training is the focus of rehabilitation treatment for patients with LBP, mainly through training the stability of core muscles to relieve symptoms and pain [4]. In recent years, the research on LBP has shifted from the degeneration of bone structure to the bone-joint-soft tissue system, and it is considered that the reduction of lumbar balance and lumbar muscle strength is the main cause of nonspecific chronic LBP. Therefore, paravertebral, back, and lateral abdominal muscle strength exercises are of great significance in improving the clinical symptoms of nonspecific chronic LBP [5].

The lumbar multifidus (LM) is the main muscle group to maintain lumbar stability. LM dysfunction is closely associated with LBP [6]. LM atrophy is more closely correlated with chronic LBP than acute LBP, as indicated by the latest research [7]. Therefore, the functional training of LM is an important part of clinical treatment [8]. Various types of training, including abdominal contraction training, swallow-type low back muscle exercise, support training, and superman training, are often recommended to enhance LM mobility. These exercises are highly effective in increasing lumbar stability, which not only reduces the recurrence of LBP but also increases the functional reserve of LM [9, 10].

However, for lumbodorsal muscle exercises, swallow-type low back muscle exercise, five-point support method, and superman training all have special requirements for space and equipment, which limits the routine exercise of lumbodorsal muscles. Therefore, there is an urgent need for a simpler and more convenient way to exercise the lumbodorsal muscles without the limitation of space and equipment, which has important clinical significance for improving the function of lumbar back muscles of patients and thus alleviating LBP. This paper makes a preliminary study on the equivalence between standing back-extension and superman training of LM, in order to find a simpler and easier way to exercise lumbodorsal muscles.

## 2. Data and Methods

### 2.1. Participants

A total of 26 healthy young volunteers admitted to Civil Aviation General Hospital from January 2018 to January 2021 were included, including 14 males and 12 females, with an age of 22-44 years (average: 31.77 ± 7.06 years), a height of 154-178 cm (average: 168.77 ± 7.14 cm), a weight of 51.5-88 kg (average: 64.65 ± 9.49 kg), and a body mass index (BMI) of 20.28-27.77 kg/m^2^ (average: 22.54 ± 1.82 kg/m^2^) (Table 1). All volunteers signed the informed consent and volunteered to participate. The inclusion criteria were as follows: no back pain in the past 6 months, ability to train for the study, BMI < 30 kg/m^2^, and no other defects. This study was approved by the Hospital Ethics Committee of Civil Aviation General Hospital.

### 2.2. Ultrasonography

A 2.5-6 MHz probe was used to measure the thickness of the LM of the left transverse process of the L5 vertebra. The subjects lay prone on the bed with a pillow on the abdomen to keep the lumbar spine straight. At rest, the thickness of the LM muscle was measured, and the lumbosacral angle was maintained at 10° or less.

### 2.3. Superman Training for Low Back Muscles

For static prone decubitus, stay horizontal prone, quiet and relaxed. For prone superman, lie down horizontally, with both shoulders and upper limbs stretched out beside the ears, and the neck, chest, and waist actively stretched to the limit; lift the hips and contract the anus, and keep the lower limbs flat together for 5 seconds. The schematic diagram of prone superman is shown in Figure 1.

### 2.4. Standing Back-Extension Exercise

For static standing, stand upright and relax. For standing back-extension, stand upright, with the upper limbs of the shoulders drooping naturally, and the upper part of the torso the same as “prone superman”; stand upright, with chin up and chest out and shoulders in horizontal position, and externally rotate both shoulders to the maximum; stretch the neck back as far as possible, straighten the waist and lift the hips, and keep the neck and lower back muscles tense. See Figure 2 for the schematic diagram of standing back-extension exercise.

### 2.5. Outcome Measures

After the subjects received superman training and standing back-extension exercise, the corresponding LM thickness of static standing and static prone decubitus and that of standing back-extension and prone superman training were compared, respectively.

### 2.6. Statistical Processing

SPSS 22.0 was the statistical software used for analysis. The quantitative variables were recorded as Mean ± SD, and the comparison between groups was made by *t*-test; the categorical variables described as percentages (%) were compared using the *χ*^2^ test. Any differences with *P* < 0.05 were considered statistically significant.

## 3. Results

### 3.1. Comparison of the Thickness of the Left LM of the Transverse Process of the L5 Vertebra between Static Standing and Static Prone Decubitus

There was no significant difference in the left LM thickness of the transverse process of the L5 vertebra between static standing and static prone decubitus (*P* > 0.05, Figure 3).

### 3.2. Comparison of the Thickness of the Left LM of the Transverse Process of the L5 Vertebra between Standing Back-Extension and Prone Superman

There was no significant statistical difference in the left LM thickness of the transverse process of the L5 vertebra between standing back-extension and prone superman (*P* > 0.05, Figure 4).

For the thickness of the left LM of the transverse process of the L5 vertebra, there was no statistical difference between static standing position and static prone decubitus position (*P* > 0.05) and between standing back-extension and prone superman (*P* > 0.05), indicating that for the training of LM, standing back-extension exercise and prone superman training are equivalent in static and dynamic conditions.

## 4. Discussion and Conclusion

Clinical studies have found that patients with LBP usually experience lumbar muscle atrophy, abnormal motor control ability, and changes in multifidus contraction pattern [11, 12]. In a previous study, pain disappeared in LBP patients after 4 weeks of treatment or exercise control, but the return of LM symmetry was only seen in those who received exercise control for 4 to 10 weeks [13]. In clinical practice, all kinds of lumbar stability exercises are used to treat LM muscle dysfunction, among which superman training is indicated in most electromyography (EMG) studies to be effective in activating LM muscle [14, 15].

In 1992, Panjabi, a renowned biomechanical scholar, proposed the following three subsystems to maintain lumbar stability [16]: for passive subsystem, it covers bones, ligaments, intervertebral discs, fascia, etc., to provide endogenous stability; for active subsystem, it includes core muscle groups and tendons to provide exogenous stability; for neural subsystem, it uses neural circuits to control the timing, sequence, and intensity of muscle contractions. The three subsystems of lumbar stability have been widely recognized, especially the core muscle, which is the most important component of the passive subsystem and has received more and more attention in recent years. The muscles around the spine constitute an exogenous balance, and the pressure in ligaments and intervertebral discs constitutes an endogenous balance. If the endogenous system is unbalanced and the surrounding muscles are strong enough, the exogenous system can still be compensated to ensure people's daily activities. If the muscle strength decreases and the exogenous system is out of balance that cannot be compensated, the stability of the lumbar spine will decline, resulting in persistent LBP. In order to avoid pain, people consciously limit their activities, which gradually leads to a further loss of muscle strength and consequently a further decline in the lumbar spine's ability to maintain balance, thus forming a vicious circle. The lumbar spine is the part with the largest load bearing, the largest range of motion, and the highest activity frequency in all stages of the spine. The coordination of lumbar bone structure with the muscle and nerve conduction system is an important guarantee for lumbar spine to exert its physiological characteristics. Hodges and Richardson [17] believed that the lumbar spine itself lacked stability and relied on the strength of muscles around the waist in the exogenous system to balance it.

The core muscles are those that can regulate the body's center of gravity to maintain the balance and stability of the trunk. Generally, they can be divided into two groups. The first is the deep core muscles, also known as local stabilizing muscles, which include transverse abdominis muscle, multifidus muscle, obliquus internus abdominis, and quadratus lumborum. The second is superficial core muscles or global stabilizing muscles, including rectus abdominis, obliquus internus abdominis, obliquus externus abdominis, erector spinae, quadratus lumborum, and gluteal muscle. A growing number of studies have shown that the coordination of these two groups of muscles maintains the stability of lumbar spine during activities of daily living [18]. Therefore, the stability of the spine and trunk will be reduced when the three subsystems or the core muscles are damaged. At present, it is believed that LBP are mainly attributed to two reasons: (1) There is dysfunction in the passive subsystem of the spine; (2) the inhibition of the function of the deep core muscles and the abnormal movement control result in the loss of the function of stabilizing and protecting the spine, plus that the function of the core muscles will not recover with the disappearance of LBP symptoms.

The so-called core stability means that when the body is completing certain sports or high-load activities, it can well control the trunk and pelvis and transfer the strength from the trunk to the limbs in an optimal way, so that the sports performance and posture can reach the best level [19]. Stability training for core muscles can reduce pain and disability, restore and enhance the muscle function of the core muscle group such as LM, promote trunk stability, and reduce the risk of injury [20]. The core muscle stability training has been proved to be effective in clinical practice in the treatment of LBP. It can not only treat LBP but also effectively increase the muscle thickness of transversus abdominis and LM and improve the proprioception and balance of subjects [21]. Therefore, core muscle stability training is of great significance to the rehabilitation of LBP.

The multifidus muscle is part of the paravertebral muscle, which lies deep and is covered by shallow erector spinae, both of which play a role in stabilizing the spine at the back and both sides of the spine. The degree of paravertebral muscle rigidity is closely related to LBP. The morphologic changes associated with LM pain have been clinically demonstrated and can be significantly alleviated with appropriate exercise training. Stability training is mainly recommended for patients with LBP to improve strength, endurance, and control of trunk muscles [22].

This study showed that there was no significant difference in the left LM thickness of the transverse process of the L5 vertebra between static standing and static prone decubitus (*P* > 0.05). Nor was there any statistical difference between standing back-extension and prone superman (*P* > 0.05). This shows that for LM exercise, standing back-extension exercise is equivalent to prone superman training in static and dynamic conditions. Therefore, in clinical work, patients with LBP can be recommended to exercise the lumbodorsal muscles by static standing and standing back-extension. The innovation of this study is to confirm that the standing back-extension exercise, as a simple exercise form that breaks through the limitations of space and equipment, is equivalent to superhuman training, which provides a new option to exercise the lumbar multifidus and relieve LBP. There are also shortcomings in this study. The sample size of this study is small, which needs to be expanded in the future to make the results more convincing. In addition, the participants of this study were all young healthy volunteers. In future studies, it is necessary to exercise LM by standing back-extension and static standing in patients with LBP and compare it with superman training, so as to make the conclusions more credible. Therefore, the sample size should be increased in the future, and the thickness of LM muscle after exercise in patients with LBP should be measured at the same time to test whether the two exercise methods are not significantly different and are equivalent.

## 5. Conclusion

In conclusion, there was no significant statistical difference in the left LM thickness of the L5 transverse process measured by ultrasonography during static standing and standing back-extension, compared with that during static prone decubitus and prone superman, respectively, indicating that the two are equivalent, which provides a simpler and more feasible method to exercise the lumbodorsal muscles for clinical practice.

## Figures and Tables

**Figure 1:** Superman training for low back muscles.

**Figure 2:** Standing back-extension exercise.

**Figure 3:** Comparison of left multifidus muscle thickness (cm) of the transverse process of the L5 vertebra between static standing and static prone decubitus.

**Figure 4:** Comparison of left multifidus muscle thickness (cm) of the transverse process of the L5 vertebra between standing back-extension and prone superman.

**Table 1:** Baseline data of subjects.

Variables	*n*	Mean ± SD
Age (years)	26	31.77 ± 7.06
Height (cm)	26	168.77 ± 7.14
Weight (kg)	26	64.65 ± 9.49
BMI (kg/m^2^)	26	22.54 ± 1.82

## Data Availability

The labeled datasets used to support the findings of this study are available from the corresponding author upon request.

## References

[1] Frymoyer J. W. (1988). Back pain and sciatica. *The New England Journal of Medicine*.

[2] Borenstein D. (1991). Low back pain. *Current Opinion in Rheumatology*.

[3] Koes B. W., van Tulder M., Lin C. W., Macedo L. G., McAuley J., Maher C. (2010). An updated overview of clinical guidelines for the management of non-specific low back pain in primary care. *European Spine Journal*.

[4] Hestbaek L., Leboeuf-Yde C., Manniche C. (2003). Low back pain: what is the long-term course? A review of studies of general patient populations. *European Spine Journal*.

[5] Verbrugghe J., Hansen D., Demoulin C., Verbunt J., Roussel N. A., Timmermans A. (2021). High intensity training is an effective modality to improve long-term disability and exercise capacity in chronic nonspecific low back pain: a randomized controlled trial. *International Journal of Environmental Research and Public Health*.

[6] MacDonald D., Moseley L. G., Hodges P. W. (2009). Why do some patients keep hurting their back? Evidence of ongoing back muscle dysfunction during remission from recurrent back pain. *Pain*.

[7] Goubert D., Oosterwijck J. V., Meeus M., Danneels L. (2016). Structural changes of lumbar muscles in non-specific low back pain: a systematic review. *Pain Physician*.

[8] Freeman M. D., Woodham M. A., Woodham A. W. (2010). The role of the lumbar multifidus in chronic low back pain: a review. *PM R*.

[9] Hides J. A., Jull G. A., Richardson C. A. (2001). Long-term effects of specific stabilizing exercises for first-episode low back pain. *Spine*.

[10] Kim C. R., Park D. K., Lee S. T., Ryu J. S. (2016). Electromyographic changes in trunk muscles during graded lumbar stabilization exercises. *PM & R : The Journal of Injury, Function, and Rehabilitation*.

[11] Danneels L. A., Coorevits P. L., Cools A. M. (2002). Differences in electromyographic activity in the multifidus muscle and the iliocostalis lumborum between healthy subjects and patients with sub-acute and chronic low back pain. *European Spine Journal*.

[12] Wong A. Y., Parent E. C., Funabashi M., Kawchuk G. N. (2014). Do changes in transversus abdominis and lumbar multifidus during conservative treatment explain changes in clinical outcomes related to nonspecific low back pain? A systematic review. *The Journal of Pain*.

[13] Hides J. A., Richardson C. A., Jull G. A. (1996). Multifidus muscle recovery is not automatic after resolution of acute, first-episode low back pain. *Spine*.

[14] Ekstrom R. A., Osborn R. W., Hauer P. L. (2008). Surface electromyographic analysis of the low back muscles during rehabilitation exercises. *The Journal of Orthopaedic and Sports Physical Therapy*.

[15] Oliver G. D., Stone A. J., Plummer H. (2010). Electromyographic examination of selected muscle activation during isometric core exercises. *Clinical Journal of Sport Medicine*.

[16] Panjabi M. M. (1992). The stabilizing system of the spine. Part i. Function, dysfunction, adaptation, and enhancement. *Journal of Spinal Disorders*.

[17] Hodges P. W., Richardson C. A. (1996). Inefficient muscular stabilization of the lumbar spine associated with low back pain. A motor control evaluation of transversus abdominis. *Spine*.

[18] Khanzadeh R., Mahdavinejad R., Borhani A. (2020). The effect of suspension and conventional core stability exercises on characteristics of intervertebral disc and chronic pain in office staff due to lumbar herniated disc. *Archives of Bone and Joint Surgery*.

[19] Lee K. (2021). The relationship of trunk muscle activation and core stability: a biomechanical analysis of pilates-based stabilization exercise. *International Journal of Environmental Research and Public Health*.

[20] Zheng Y., Ke S., Lin C. (2019). Effect of core stability training monitored by rehabilitative ultrasound image and surface electromyogram in local core muscles of healthy people. *Pain Research & Management*.

[21] Hlaing S. S., Puntumetakul R., Khine E. E., Boucaut R. (2021). Effects of core stabilization exercise and strengthening exercise on proprioception, balance, muscle thickness and pain related outcomes in patients with subacute nonspecific low back pain: a randomized controlled trial. *BMC Musculoskeletal Disorders*.

[22] Hebert J. J., Le Cara E. C., Koppenhaver S. L. (2020). Predictors of clinical success with stabilization exercise are associated with lower levels of lumbar multifidus intramuscular adipose tissue in patients with low back pain. *Disability and Rehabilitation*.

